# An Easy Path for Correlative Electron and Super-Resolution Light Microscopy

**DOI:** 10.1038/s41598-019-52047-2

**Published:** 2019-10-29

**Authors:** Dorothea Pinotsi, Simona Rodighiero, Silvia Campioni, Gabor Csucs

**Affiliations:** 1 Scientific Center for Optical and Electron Microscopy, ETH Zurich, Zurich, Switzerland; 2 Present Address: European Institute of Oncology, Department of Experimental Oncology, Milan, Italy; 3 Department of Health Sciences and Technology, ETH Zurich, Zurich, Switzerland; 4 Present Address: Laboratory for Cellulose and Wood Materials, EMPA, Dübendorf, Switzerland

**Keywords:** Nanoscale biophysics, Microscopy

## Abstract

A number of new Correlative Light and Electron Microscopy approaches have been developed over the past years, offering the opportunity to combine the specificity and bio-compatibility of light microscopy with the high resolution achieved in electron microscopy. More recently, these approaches have taken one step further and also super-resolution light microscopy was combined with transmission or scanning electron microscopy. This combination usually requires moving the specimen between different imaging systems, an expensive set-up and relatively complicated imaging workflows. Here we present a way to overcome these difficulties by exploiting a commercially available wide-field fluorescence microscope integrated in the specimen chamber of a Scanning Electron Microscope (SEM) to perform correlative LM/EM studies. Super-resolution light microscopy was achieved by using a recently developed algorithm - the Super-Resolution Radial Fluctuations (SRRF) - to improve the resolution of diffraction limited fluorescent images. With this combination of hardware/software it is possible to obtain correlative super-resolution light and scanning electron microscopy images in an easy and fast way. The imaging workflow is described and demonstrated on fluorescently labelled amyloid fibrils, fibrillar protein aggregates linked to the onset of multiple neurodegenerative diseases, revealing information about their polymorphism.

## Introduction

The development of correlative Light and Electron Microscopy (LM and EM) methods has contributed to significant advances in the understanding of biological, chemical and physical processes^1–5^. With such methods one can harvest the advantages of both fields of microscopy: electron microscopy provides the highest level of detail in structural information, with resolution down to the nanometer level. On the other hand, light microscopy provides chemical specificity, is typically less-invasive and potentially allows live imaging. However, light microscopy is clearly limited in resolution compared to electron microscopy. This “traditional” limit (caused by the diffraction of light) has been overcome in the last years by the development of optical super-resolution microscopy techniques, such as STORM, PALM, SIM and STED^6–9^. Some of these techniques can reach a resolution limit down to tenths of nanometers. It is clear that a synergic combination of super-resolution LM combined with various forms of EM could lead to unprecedented information on the process under study. Often however, such approaches are based on protocols which are complex and very difficult to implement and require transferring of the sample between different setups, the use of patterned substrates^10,11^, as well as rigorous image analysis algorithms for image alignment and correlation^12–15^. Moreover, these methods are time-demanding and costly, as they require the availability of expensive setups.

Here, we present a simple approach to perform correlative super-resolution light and electron microscopy using a Scanning Electron Microscope (SEM) system equipped with fluorescence capabilities. The simplicity of the method we describe is based on: (a) the commercial availability of a wide-field fluorescence microscope that can be mounted inside an SEM chamber and (b) the application of a recently developed algorithm called Super Resolution Radial Fluctuations (SRRF) for simple and cost-effective super-resolution light microscopy^16^. This method can be performed with a standard wide-field fluorescent microscope and solely uses an ImageJ plugin for the image analysis (requiring a time-lapse acquisition of the field of view of interest).

As an example application demonstrating the value of our approach, we studied the morphology of dual-color labeled amyloid fibrils formed by the human α-Synuclein (α-Syn) protein, whose aggregation is related to the onset of Parkinson’s disease^17,18^. Amyloids are nanoscale filaments (typically 2–10 nm wide and up to 10 μm long, depending on the aggregation conditions) that are of high scientific interest not only because of their relation to human diseases, but also because nowadays non-pathological amyloid-like fibrils can be formed *in vitro* from small peptides and used for technological purposes^19,20^. A detailed characterization of the properties of these aggregates is often hampered by their small size, their polymorphism (i.e. one protein/peptide precursor can give rise to different types of fibrils, often co-existing within the same sample), and by difficulties in chemically distinguishing different segments within an aggregate. We applied our method to the analysis of α-Syn fibrils obtained from seeded experiments, where short fibers called “seeds” were used to initiate the aggregation of monomeric α-Syn, and we made use of a previously published dual-color approach to distinguish the original “seed” from the elongating part^21^. The obtained results show that with our approach we are able not only to distinguish the “seed” units from the elongating monomers incorporated in the fibers, but also to identify details on the filaments that are involved in the bundles.

## Results

Amyloid fibrils are highly ordered, filamentous structures that form through a complex aggregation pathway, and have a high tendency to interact with each other forming small bundles, sheets and eventually plaques. Their properties and their mechanism of formation have been investigated using various imaging techniques: EM, AFM and super-resolution microscopy among others^22,23^. Recently, single-molecule localization microscopy has been used in different studies in order to probe the morphology of protein aggregates both *in vitro* and *in situ*, in cells^24^.

In our experiments, we have covalently attached a fluorescent dye to the α-Syn protein chain, in order to produce labeled fibrils (see Materials and Methods for details on fibril preparation). As compared to immunofluorescence staining, site-specific labeling of α-Syn allows probing the morphology of the aggregates more directly, because of the small size of the fluorescent dye which is linked to the protein. We visualized the process of fibril elongation using a “seeded” aggregation assay^21,25–27^, where we mixed a solution of preformed, small fibrils (“seeds”) of α-Syn labeled with Alexa Fluor 568 (AF568), with a second solution containing α-Syn in its monomeric state with 10% of the protein molecules labeled with Alexa Fluor 647 (AF647). This was added to the preformed α-Syn seeds solution at a 10-fold excess (by molarity), giving rise to the dual-color labeled fibrils.

Figure 1 depicts schematically the method workflow from protein fibril preparation to the overlaid super-resolution and SEM images. The first step is the protein fibril preparation, as described previously^21^. Subsequently, a drop of 10 μl of the sample solution is deposited on a commercially available indium tin oxide (ITO)-coated glass coverslip. The solution is left to adsorb for approximately 30 min. Next, the coverslip is washed at least 5 times with distilled water, followed by a drying procedure with nitrogen flow. The coverslip is then ready to be mounted into the SEM chamber. First, the fluorescence signal is used to focus at the sample with the objective of the optical microscope. The electron beam is then focused on the sample surface and adjusted performing the aperture alignment, astigmatism correction and fine focusing. At this point, the software-integrated alignment procedure allows to precisely align the optical field of view with the SEM field of view^28^.

**Figure 1:** Method workflow. (**a**) Protein fibril preparation (see text for details, schematic reprinted (adapted) with permission from^21^ https://pubs.acs.org/doi/abs/10.1021/nl4041093. Copyright 2013 American Chemical Society). (**b**) A drop of 10 μl of the protein fibrils is deposited on an ITO-coated glass coverslip, the solution is left to adhere for approximately 30 min, washed 5 times with distilled water, and dried with a nitrogen gun. (**c**) The ITO-coated glass coverslip is loaded in the SEM chamber and the chamber is evacuated. After the alignment of the fluorescence/SEM fields of view, a 2-channel time-lapse acquisition (200 images) is performed followed by the SEM image acquisition. The fluorescence image stack and the SEM image are saved and the former is used for applying the SRRF algorithm. The super-resolution image is then merged with the SEM image.

After the alignment of the optical and the SEM fields of view, a time-lapse acquisition for each of the two excitation wavelengths for the AF568, shown in green, and the AF647 shown in red, is performed with an sCMOS camera. For SRRF reconstruction, an image stack (time-lapse acquisition) consisting of 200 images is needed. After this step a SEM image of a smaller area which covers the central part of the sCMOS field of view (FOV) is taken. The fluorescence image stack and the SEM image are saved and the former is then processed with the SRRF algorithm, as described below.

This correlative microscopy workflow required that the optical images were acquired in the same vacuum conditions as the SEM images. We acquired both fluorescence and SEM images in high vacuum (approximately 5 m Pa). It is known that fluorescent proteins (FP) have decreased quantum yields in vacuum compared to ambient pressure^29^, so we tested the Alexa dyes at different sample chamber pressures to check if they experience a similar decrease in quantum yield in vacuum as the FP. We acquired the emitted fluorescence under identical excitation powers and camera exposure times of commercially available beads (TetraSpecks, Invitrogen) labelled with 4 different Alexa dyes (A405, A488, A561, A647) in HV (5 m Pa), at 50 Pa, 100 Pa and 240 Pa exploiting the Variable Pressure mode of the SU5000 SEM with a 40x/0.95 objective lens. We did not observe a clear trend of the emitted fluorescence vs the sample chamber pressure. Even if we consider that the higher pressure in the SEM chamber (240 Pa) is a very low pressure in comparison to the ambient (≈100 kPa), the emitted fluorescence going from 240 Pa to 5 mPa didn’t change dramatically (A405 from 9513 ± 273 counts to 9941 ± 230; A488 from 9205 ± 315 to 9769 ± 337; A568 from 9397 ± 248 to 10013 ± 212; A647 from 9340 ± 255 to 10000 ± 214, at 240 Pa and HV, respectively), suggesting a different behavior of Alexa dyes in vacuum with respect to the fluorescent proteins, at least in our experimental conditions.

To choose the proper SEM parameters to visualize the α-Syn fibrils, different acceleration voltages, dwell times and pixel sizes were used. The Z position of the sample stage was fixed to a certain height considering the steric constraints between the SEM objective lens and the stage itself, allowing a working distance range (WD) between 11.6 and 11.8 mm, depending on the beam parameters. In Fig. 2a set of SEM images of fibrils acquired with different parameters are shown. From (a) to (e) only the acceleration voltage (V_acc_) has been modified. At 2 kV (a) and 5 kV (b) it is difficult to distinguish the fibrils on the ITO substrate, due to the poor resolution at this low V_acc_ and long WD. The fibrils’ visibility improves at 10 kV (c) and becomes optimal at 20 (e) and 30 kV (f). Imaging the fibrils with high acceleration voltage gave good resolution images, but we cannot exclude that a certain amount of radiation damage directly caused by the electron beam and probably thermal effect was produced by the imaging itself, together with the carbon contamination of the sample surface. We actually observed that after 2 or 3 SEM acquisitions the fibrils disappeared (not shown). We hypothesized that both beam-induced contamination and beam damage, which scale with the energy deposited on the sample, could have an impact on the image contrast of the fibrils imaged on the ITO coated coverglass.

**Figure 2:** SEM image optimization. SEM imaging of the amyloid fibrils on the ITO-coated coverslip performed at different acceleration voltages (V_acc_), pixel sizes and pixel dwell times, respectively: (**a**) 2 kV, 3.4 nm, 10 μs; (**b**) 5 kV, 3.4 nm, 10 μs; (**c**) 10 kV, 3.4 nm, 10 μs; (**d**) 20 kV, 3.4 nm, 10 μs; (**e**) 30 kV, 3.4 nm, 10 μs; (**f**) 30 kV, 6.8 nm, 40 μs; (**g**) same parameters as in (**f**); in (**h**,**i**) the two insets shown in panel (g) have been digitally magnified to highlight a branch, panel (h), and two overlapping fibrils, panel (i). The working distance was between 11.8 and 11.6 mm in all images and the scale bar is 600 nm in panels (a–g) and 150 nm in panels (h,i).

Doubling the pixel size and keeping the same scan frame time (42 s) improved the contrast of the fibrils with respect to the background signal (f). This was obtained by reducing the number of pixels from 2048 × 2048 to 1024 × 1024 and increasing the dwell time from 10 μs to 40 μs. In this way, the total energy provided to the sample during imaging didn’t change, and we didn’t expect a different contamination or beam damage effect. On the other hand however, on a pixel basis, the increased dwell time resulted in a more efficient signal collection, especially from the ITO substrate, which resulted in a brighter background with respect to the α-syn fibrils which are mainly composed by carbon. In all the subsequent acquisitions these parameters have been used. In (g) another set of fibrils is shown and the selected areas in the h and i regions of interest (ROIs) are magnified in panels (h) and (i) where fibril branching and two overlapping fibrils are shown, respectively.

In Fig. 3 we show the application of the method and the correlative imaging of dual-color labeled protein fibrils of α-Syn, on an ITO coated glass coverslip. Figure 3a is the conventional wide-field image of the fibrils, where the red and the green fluorescence cannot be discerned due to the diffraction limit. Figure 3b shows the corresponding SEM image of the same protein fibrils. In the magnified views shown in panels b_1_ and b_2_, one can observe that the fibrils in these areas consist of two filaments that overlap with each other. In panel b_1_ the two fibrils are twisted, forming a helix. It is also visible that one of the two fibrils has a “wavy” morphology. This feature could be due to the helicity reported for amyloid fibrils^30^, again showing the extent of morphological detail that can be obtained only with the SEM imaging.

**Figure 3:** Correlative imaging and WF and SRRF resolution comparison. (**a**) Wide-field fluorescence image of the Alexa 568 (green) and Alexa 647 (red) signals of amyloid fibrils. (**b**) SEM image of the protein fibrils shown in (**a**). b_1_ and b_2_ are the two magnified views of the corresponding areas drawn in (**b**). (**c**) Super-resolved SRRF image of the same fluorescent fibrils. (**d**) Overlay of the SRRF image shown in c and the SEM shown in (**b**). d_1_ and d_2_ are the two magnified views of the corresponding areas drawn in (**b**,**d**). Scale bar: 800 nm in (**a**–**d**) and 150 nm in b_1_, b_2_, d_1_, d_2_. (**e**) SRRF processed image of a fibril (green channel) and (**f**) corresponding wide-field image. Scale bar: 800 nm. In (**g**) the Gaussian fits of the normalized intensity profiles along the red and blue lines shown in e and f are shown.

In Fig. 3c we show the super-resolved SRRF image of the same fluorescent fibrils, where we can clearly distinguish between the differently labeled parts of the fibrils: the part that corresponds to the initial “green” seed and the part that stems from the “red” monomeric protein. The overlay of the SRRF image and the SEM, shown in Fig. 3d enables us to correlate the structure of the fibrils (from the SEM) and the fluorescence signal. The magnified views in panels d_1_ and d_2_ are the overlays of the SEM images with the corresponding super-resolved SRRF images. In panel d_1_ a green seed at the top left of the fibril is intertwisted with a red fibril. Differently from the red fibril, the green seed has a ‘wavy’ structure. In panel d_2_ a red fibril is overlapping with a green seed, with a less visible but still discernible ‘wavy’ structure, which will be discussed below.

Two magnified views of the super-resolved SRRF and of the wide-field image of a green seed are shown in Fig. 3e,f, respectively. In panel (g) the plotted intensity cross section profiles along the red and the blue line shown in (e) and (f) were normalized and fitted with a Gaussian function, to calculate the full-width-half maximum (FWHM) in each case. The improvement in resolution in the processed SRRF image is evident. The FWHM of the fibril obtained from the super-resolution SRRF image is around 60 nm (versus 350 nm obtained from the conventional fluorescence image) which is much closer to the true value of the FWHM of the amyloid fibrils, including the fluorescent dye.

## Discussion

It is interesting to point out that thanks to the SEM resolution, which is in the same range as the fibrils’ cross section (few nanometers), one can clearly visualize overlapping fibrils, and the overlay with the super-resolved SRRF fluorescent images that bring the information of the specific labeling, allows distinguishing between seeds and polymerized “red” monomers, even though the resolution of the fluorescent image is limited (around 60 nm for SRRF vs 350 nm for conventional fluorescence microscopy). Furthermore, we suggest that the observed “wavy” structures of some amyloid fibrils may originate from two different effects: first, one reason may be the method of preparation used. The first part of our fibril preparation protocol (the elongation of unlabeled seeds with green fluorescent molecules) was done under agitation in an orbital shaker (Thermomixer) in order to prepare short fibrils, while the second part of the process (the elongation of green seeds with the red color) was in quiescent conditions (see Methods) in order to monitor the growth of the green seeds under more physiologically relevant conditions. As also suggested by other reports^31,32^ vortex and shear flow can induce the formation of entangled bundles of fibers.

Secondly, it is highly common for amyloids to show polymorphism and α-syn fibrils have been shown to change morphology over time. Therefore, a different stage of maturation and polymorphism may also be responsible for the difference between the seed region and the remaining portion of the fiber^33^.

We thus present a correlative SEM and optical super-resolution microscopy method that compared to other approaches is fast, does not require sample transfer, patterned substrates, fiducials and specific image registration software. On the contrary, it can be performed practically at any type of SEM that can allow for an integrated wide-field fluorescent microscope, without the need for expensive lasers. Nevertheless, we also note that there are specific pitfalls in our method, compared to other approaches which use separate electron microscopy and super-resolution setups: the most important limitation is that the method we present is not compatible with live-cell fluorescent imaging. Furthermore, *in vitro* samples or other specimens such as amyloid fibrils are optimally suited for this methodology, as they do not require electron microscopy preparation methods (such as fixations) which would in turn endanger the preservation of the fluorescent labels. We also point out that because of the increase in resolution thanks to the SRRF algorithm, a possible misalignment between different fluorescent channels should be taken into account, especially when, differently from our filter configuration, a multiband beam splitter is used in combination with a motorized emission filter wheel. The mechanical movement of the filters can lead to image shifts on the order of 10–50 nm and this could introduce a possible source of error in the overlay of the fluorescence channels that should be considered in that case. Additionally, even though patterned substrates are not required, there is still the need for conductive ones- in our case we used ITO coated coverslips. Finally, due to the stage constraints of the integrated wide-field microscope, the working distance for the SEM is fixed, which could eventually decrease the achieved SEM resolution.

In conclusion, we present a simple and relatively cost-effective approach to perform correlative electron and optical super-resolution microscopy. Thanks to the described workflow, we were able to easily discern details of the amyloid fibril aggregation and morphology. The super-resolution fluorescence image formed via combining the SRRF algorithm with a standard wide-field fluorescence microscope allowed us to identify and distinguish between the original seed fibrils and the elongation/polymerized part. In addition, the SEM image allowed us to discern in detail how these two parts interact with each other: if there is for example fibril overlap, branching or intertwisting of filaments. We plan to continue this experimental approach to gain further insights into how different aggregation conditions can affect the mechanistic and structural details of the aggregation and fibril self-assembly processes, which is of high interest for research on amyloid protein aggregation kinetics.

## Methods

### α-Syn protein preparation and labeling

Recombinant human α-Syn was produced as previously described^25^. For labeling, a mutant of α-Syn having a single Cysteine (Cys) residue inserted at the C-terminal of the protein (α-Syn-C141) was prepared. The position was chosen for not to interfere with the aggregation process of the protein. Since wild-type α-Syn does not contain any Cys, the insertion of an individual Cys allowed, using site-directed labeling strategies, to include a single label molecule on each protein chain. The mutant was expressed and purified as described^25^, with addition of 2 mM dithiothreitol to the purification buffers, to prevent disulfide bond formation during the purification process. At the end of the process, all samples were extensively buffer exchanged and concentrated in Milli-Q water by ultrafiltration, using an Amicon Stirred cell with a 5 kDa molecular weight cut-off membrane (Merck Millipore, MA, USA); and they were stored at −25 °C as lyophilized powder until use.

Alexa Fluor dyes (Fisher Scientific AG, Reinach, Switzerland) were first dissolved in dimethyl sulfoxide at 10 mM concentration, aliquoted, and kept frozen and in the dark. Aliquots of α-Syn-C141 (10 mg) were dissolved in 1 ml of 10 mM sodium phosphate buffer, pH 7, with 0.05% sodium azide and tris(2-carboxyethyl)phosphine was immediately added at a 1:1 molar ratio with the protein, as this reducing agent does not affect the conjugation with maleimide-reactive dyes. After mixing all components, the pH was adjusted to 7.3 with 1 M sodium hydroxide. For labelling, either Alexa Fluor 568 (AF568) or Alexa Fluor 647 (AF647) where mixed with an aliquot of the protein sample at a 1:2 protein:dye molar ratio. The samples where then incubated in the dark at room temperature for 2 h, followed by overnight incubation at 4 °C. Subsequently, the excess of dye was then removed by desalting using a 5 ml HiTrap desalting column (GE Healthcare, IL, USA) equilibrated with water, followed by prolonged dialysis against water. Mass spectrometry and amino acid analysis were then used to verify the molecular weight of the final product and the protein concentration of the labeled samples.

### α-Syn fibril preparation

Lyophilized aliquots of unlabeled α-Syn were first dissolved in 10 mM sodium phosphate buffer, pH 7, with 0.05% sodium azide at a protein concentration of 2 mM. Such highly concentrated samples are usually turbid and their pH needs to be re-adjusted to 7 with small additions of 1 M sodium hydroxide, for the protein to fully dissolve. The sample was then dialysed overnight at 4 °C against a high excess (1:1000 volume ratio) of 10 mM sodium phosphate buffer, pH 7, with 0.05% sodium azide. On the following day, residual protein aggregates were eliminated by filtration with a 100 kDa molecular weight cut-off centrifugal filter (Amicon Ultra 100 kDa from Merck Millipore, MA, USA) and the final concentration of the sample was determined by ultraviolet-visible absorbance, using an extinction coefficient of 5960 M^−1^ cm^−1^ (calculated with Protparam).

First, unlabeled fibrils were obtained by incubating samples at 300 μM concentration in the same sodium phosphate buffer for one week, at 37 °C and on a rotating device. Non-binding 1.5 ml microcentrifuge tubes from Eppendorf (Hamburg, Germany) were used. These unlabeled fibrils were then sonicated with a tip sonicator to reduce their size using the following parameters: 20% tip power, alternating cycles of 2.0 s of sonication and 0.5 s break, for a total duration of 30 min of sonication. To prevent over-heating, the tube containing the sample was floating on a large water-bath (ca. 1.8 L) with room-temperature water. Sonicated, unlabeled seed fibrils were used to promote the aggregation of a mixture of monomeric unlabelled α-Syn (90%) and labelled with AF568 (10%). The total seeds concentration was 3 μM (monomer equivalents). The total concentration of the monomeric protein was 150 μM. After three days of incubation at 37 °C on an Eppendorf Thermomixer with 500 rpm orbital shaking, fibers giving green fluorescence were obtained. Finally, these AF568 labelled fibers (diluted to 5 μM) were used to promote the aggregation of a mixture of monomeric unlabeled α-Syn (90%) and labelled with AF647 (10%), at a total monomeric protein concentration of 50 μM. The samples were then incubated at 37 °C under quiescent conditions for 4 days.

### Scanning electron microscopy and correlative microscopy

The correlative microscopy imaging was performed with an integrated microscope which allowed simultaneous observation of a sample area with both fluorescence microscopy and scanning electron microscopy (SEM). The Secom platform (Delmic B.V., Delft, The Netherlands) integrated in a Hitachi SU5000 Scanning Electron Microscope (Hitachi High-Technologies Europe GmbH, Krefeld, Germany) was used for fluorescence imaging.

A drop of 10 μl of the dual-color α-Syn amyloid fibril solution (5 μM in 10 mM phosphate buffer, pH = 7) was deposited on a commercial ITO coated coverglass (Optics Balzers AG, Balzers, Liechtenstein) for 30 min, washed 5 times with ddH_2_O and dried with a N_2_ gas gun. The ITO coated coverglass was then glued with carbon cement to an Aluminium support and mounted onto the Secom stage.

#### Fluorescence imaging

Wide-field fluorescence imaging was performed with a 60x/1.4NA oil immersion objective (Nikon Instruments Europe BV, Amsterdam, Netherlands). The AF568 and AF647 dyes were excited with the 561/14 nm and 631/28 nm channels of an LED light source (Lumencor, Beaverton, Oregon, USA), respectively. A multiband dichroic mirror was used (Di01-R405/488/561/635–25 × 36, Semrock) and the emitted fluorescence passed through a quad-band bandpass filter (FF01-440/521/607/700-25, Semrock). The fluorescence signal was acquired with a Zyla 4.2 sCMOS camera with sensor size of 2048 × 2048 pixels and a pixel size of 6.5 μm (Andor Technology Ltd., Belfast, UK). The correct positioning and focusing of the samples were first performed at ambient pressure, then the SEM chamber was evacuated and the fluorescence microscopy and the SEM imaging were performed at least 2 hours later, to allow the outgassing of the vacuum compatible immersion oil (Delmic). The sample was then refocused and an area for SEM/fluorescence alignment was chosen. The goal of this alignment procedure is to ensure that the axes of the optical lens and the e^−^ beam are aligned and it is done in two-steps: first, exploiting the cathodoluminescence signal produced by the e^−^ beam-glass interaction, the optical field of view is centered with respect to the e^−^ beam by moving the objective lens in x and y; then, an automatic fine alignment procedure of the e^−^ beam center and correction of the optical scaling with subpixel accuracy are done. These operations are performed by generating a 4 × 4 grid of e^−^ beam spots. With this grid of pointers the alignment procedure can correct for translation, scaling, rotation and possibly non-linear distortions with an accuracy better than 50 nm (fine alignment)^28^.

#### SEM Imaging

The SEM used for the experiments was equipped with a Schottky Field Emission (FE) source and an Everhart-Thornley (E-T) detector, a Back Scattered Electron (BSE) detector and a Ultra Variable-Pressure detector (UVD).

The optimization of the SEM imaging parameters was performed at a fixed beam current (approximately 1 nA), objective lens aperture, working distance (WD) and magnification (50 kX, horizontal field of view 6.95 μm) but different acceleration voltages (2, 5, 10, 20, 30 kV), dwell time (10, and 40 μs) and pixel sizes (3.4 and 6.8 nm). The Secom (Delmic) stage has a fixed Z position and all the images were acquired between 11.6 and 11.8 mm of WD. The SEM signal was collected by the E-T detector. The fibrils were completely transparent for the back scattered electron (BSE) detector (not shown).

#### Correlative microscopy imaging

The workflow for the correlative microscopy imaging is summarized in Fig. 1 and is as follows:

1. Focusing of the sample in fluorescence mode using the Z movement of the objective lens;
2. Electron beam adjustment: focusing, objective lens aperture alignment, fine focusing and astigmatism correction;
3. Alignment of the fluorescence field of view with respect to the e^−^ beam and exploiting the x,y movement of the optical objective lens^28^.
4. 2-channel sequential fluorescence time-lapse acquisition with 200 mW LED power, 500 ms exposure time, 200 frames.
5. 2-channel single fluorescence acquisition with 200 mW LED power, 2 s exposure time and SEM acquisition (30 kV acceleration voltage, 40 μs dwell time, 11.6 mm WD and 6.8 nm pixel size and 1024 × 1024 pixels) followed by the fluorescence-SEM images fine alignment^28^.

### Super-resolution microscopy using SRRF

SRRF is a purely computational super-resolution approach which is related to single molecule localization approaches, but can actually be employed also with overlapping fluorophores. This means that no blinking is required. As a result, it is applicable for any type of fluorescent dye or protein and can be used with any microscopy setup, such as wide-field, TIRF and confocal.

For SRRF imaging, the input data for the computational reconstruction is a sequential series of images of the fluorescently labeled specimen, but contrary to single molecule localization methods there is no requirement for sparsely emitting fluorophores, neither are the blinking properties of the fluorophore so important as in single molecule localization studies. SRRF is based on the assumption that the image is formed of point sources convolved with a point spread function (PSF) that displays a higher degree of local symmetry than the background. Rather than detect and localize single radially symmetric points (as it is done in single molecule localization approaches) however, for each frame in an image sequence SRRF calculates the degree of local gradient convergence (referred to as “radiality”) across the entire frame, on a sub-pixel basis. In practice, the original image is upsampled to e.g. 5 × 5 subpixels. For each subpixel, the local intensity gradients are calculated and a radiality map is created. The radiality signal of a point emitter has a singificantly smaller FWHM than its PSF, hence a significantly higher resolution can be achieved. As noise patterns can also show up in the radiality signal (and could mask the real signal), temporal analysis (based on an image sequence) can help to reduce/eliminate them. From a practical point of view our tests (in accordance with the original publication) show that approximately 200 frames are required for SRRF imaging and afterwards a new image can be computed using the SRRF Fiji plugin. The achievable lateral resolution depends on a number of factors but in our case (as discussed later) it was around 60 nm.

For more details on the mathematical and technical aspects of SRRF the reader is referred to the relevant publications^16,34^.

More specifically, each time-lapse acquisition consisting of 200 frames for each of the two fluorescence channels was background (BG) corrected. The bleed-through of the AF647 dye in the green channel was determined and the green fluorescent channel was corrected accordingly, as follows:

Briefly, AF647-only labelled α-Syn fibrils were imaged with the same acquisition parameters of the double-labelled fibrils and after BG correction the mean fluorescence intensity (I) has been calculated in more than 60 different ROIs of 4 × 4 pixels in each channel. The mean intensity of the AF568 in each ROI channel was plotted versus the mean intensity of the AF647 channel and the fraction of the AF647 signal acquired in the AF568 channel (bleed-through)- was calculated as the slope of the linear regression of the points (I_(AF568)_/I_(AF647)_ = 0.16). Afterwards, each frame (f_i_) of the AF568 channel of the double labelled time series was pixel by pixel corrected (I_(AF568corr)_ (f_i_) = I_(AF568)_ (f_i_) − 0.16 * I_(647)_ (f_i_).

The bleed-through of the AF568 dye in the red channel was negligible. The corrected time series were then processed using the ImageJ plugin provided in the NanoJ-SRRF software package (https://bitbucket.org/rhenriqueslab/nanoj-srrf/wiki/NanoJ%20sample%20data). In the user settings: a ring radius of 0.5, a radiality magnification of 7 and a number of axes in ring of 6 were applied. In the advanced settings for the temporal analysis we used the method of Temporal Radiality Pairwise Product Mean (TRPPM). The two super resolved resulting images were overlaid in ImageJ and then manually merged with the SEM image, considering the respective fields of view.

The FWHM of the intensity line profile of the fibril shown in Fig. 3e,f was calculated from the Standard Deviation (SD) of the Gaussian fitting (Y = Amplitude * exp(−0.5 * ((X-Mean)/SD)^2^) shown in Fig. 3g, as FWHM = 2.355 * SD.

As reported by the authors in^34^, the resolution of the final SRRF image will scale with the degree of fluctuations exhibited in the raw data. This can be consistently better than 150 nm^16^. Parameters that affect the resolution of the final image are the illumination intensity, the camera exposure time and the number of frames acquired and it can approach resolutions achieved by the other super-resolution techniques such as SMLM and STED. This shows that indeed this method can greatly improve the resolution especially in a live cell-context, without the need for special setups, lasers or fluorophores. In our case and the application we demonstrate the resolution was on the order of 60 nm, calculated by the FWHM of the amyloid fibrils whose real width should be less than 10 nm. This gives almost a 6-fold improvement over the wide-field resolution of ∼350 nm.

## Data availability

Additional data that support the findings of this study are available from the corresponding authors upon request. Further permissions related to the schematic in Fig. 1a should be directed to ACS.
